RETRACTED

# Mutations in the Fusion Protein Cleavage Site of Avian Paramyxovirus Serotype 4 Confer Increased Replication and Syncytium Formation *In Vitro* but Not Increased Replication and Pathogenicity in Chickens and Ducks

**DOI:** 10.1371/journal.pone.0050598

**Published:** 2013-01-14

**Authors:** Shin-Hee Kim, Sa Xiao, Heather Shive, Peter L. Collins, Siba K. Samal

**Affiliations:** 1 Virginia-Maryland Regional College of Veterinary Medicine, University of Maryland, College Park, Maryland, United States of America; 2 Experimental Transplantation and Immunology Branch, National Cancer Institute/National Institute of Health, Bethesda, Maryland, United States of America; 3 Laboratory of Infectious Diseases, National Institute of Allergy and Infectious Diseases, Bethesda, Maryland, United States of America; Texas A&M Veterinary Medical DIagnostic Laboratory, United States of America

## Abstract

To evaluate the role of the F protein cleavage site in the replication and pathogenicity of avian paramyxoviruses (APMVs), we constructed a reverse genetics system for recovery of infectious recombinant APMV-4 from cloned cDNA. The recovered recombinant APMV-4 resembled the biological virus in growth characteristics *in vitro* and in pathogenicity *in vivo*. The F cleavage site sequence of APMV-4 (DIQPR↓F) contains a single basic amino acid, at the -1 position. Six mutant APMV-4 viruses were recovered in which the F protein cleavage site was mutated to contain increased numbers of basic amino acids or to mimic the naturally occurring cleavage sites of several paramyxoviruses, including neurovirulent and avirulent strains of NDV. The presence of a glutamine residue at the -3 position was found to be important for mutant virus recovery. In addition, cleavage sites containing the furin protease motif conferred increased replication and syncytium formation *in vitro*. However, analysis of viral pathogenicity in 9-day-old embryonated chicken eggs, 1-day-old and 2-week-old chickens, and 3-week-old ducks showed that none the F protein cleavage site mutations altered the replication, tropism, and pathogenicity of APMV-4, and no significant differences were observed among the parental and mutant APMV-4 viruses *in vivo*. Although parental and mutant viruses replicated somewhat better in ducks than in chickens, they all were highly restricted and avirulent in both species. These results suggested that the cleavage site sequence of the F protein is not a limiting determinant of APMV-4 pathogenicity in chickens and ducks.

## Introduction

The family *Paramyxoviridae* consists of enveloped viruses with a nonsegmented, single-stranded, negative-sense RNA genome [1]. The family is divided into two subfamilies: *Paramyxovirinae* and *Pneumovirinae*. The subfamily *Paramyxovirinae* comprises five genera: *Rubulavirus*, *Respirovirus*, *Morbillivirus*, *Henipavirus*, and *Avulavirus*. Subfamily *Pneumovirinae* is divided into two genera: *Pneumovirus* and *Metapneumovirus*. Nearly all of the paramyxoviruses that have been isolated from avian species are classified into the genus *Avulavirus* and are called avian paramyxoviruses (APMVs); the only exceptions are the avian metapneumoviruses, which are classified in the genus *Metapneumovirus*. The APMVs of genus *Avulavirus* have been divided into nine different serotypes (APMV 1 to 9) based on hemagglutination inhibition (HI) and neuraminidase inhibition (NI) assays [2], and more recently a tenth serotype has been provisionally identified [3]. APMV-1, which comprises all strains of Newcastle disease virus (NDV), has been extensively characterized because virulent NDV strains cause severe disease in chickens and have a major economic impact. Complete genome sequences and reverse genetics systems are available for several NDV strains [4]–[8]. As an initial step towards characterizing other APMV serotypes, complete genome sequences of one or more representative strains of APMV serotypes 2 to 9 have been determined [9]–[16].

RETRACTED

The APMVs are frequently isolated from a wide variety of avian species worldwide. APMV-1 has been isolated from most species of birds and, as noted, can be highly pathogenic and has a major agricultural impact. APMV-2 and -3 also have been reported to cause significant disease in poultry [17]–[18], whereas the pathogenic potential of serotypes 4–9 is generally unknown [19]. APMV-4 strains have been isolated predominantly from feral birds of the order *Anseriformes* [20] and from domestic ducks, chickens, and geese [21]–[23]. APMV-4 has been reported to cause an increase in white-shelled eggs but did not affect the egg production in laying hens [2]. The genome of the prototype APMV-4 strain duck/Hong Kong/D3/75 consists of 15,054 nt [10], which follows the “rule of six” common to other members of subfamily *Paramyxovirinae*. APMV-4 encodes a nucleocapsid protein (N), a phosphoprotein (P), a matrix protein (M), a fusion glycoprotein (F), a hemagglutinin-neuraminidase glycoprotein (HN), and a large polymerase protein (L). The genes are flanked on either side by highly conserved transcription start and stop signals and have intergenic sequences varying in length from 9 to 42 nt. The genome contains a 55 nt leader region at the 3′ end. The 5′ trailer region is 17 nt, which is the shortest in the family *Paramyxoviridae*.

Our understanding of the viral factors responsible for tissue tropism and virulence of APMVs is incomplete and is based mainly on studies with NDV in chickens. For NDV, the amino acid sequence at the F protein cleavage site has been identified as the primary determinant of NDV pathogenicity in chickens [8], [24]. The NDV F protein, like that of all paramyxoviruses, is synthesized as a precursor (F0) that is activated by cleavage by host cell protease into two disulfide-linked subunits F2-F1 [25]. Cleavage of the F protein is necessary for virus entry and cell-to-cell fusion. The F protein of virulent NDV strains typically contains a polybasic cleavage site [(R/K)RQ(R/K)R↓F] that includes the preferred cleavage site for furin [RX(R/K)R↓], which is an intracellular protease present in a wide range of cells and tissues [26]. The F protein of these strains can be cleaved in most tissues, thus providing the potential for systemic spread. In contrast, avirulent NDV strains typically contain basic residues at the -1 and -4 positions in the cleavage site [(G/E)(K/R)Q(G/E)R↓L], lack the furin site, and depend on secreted protease (or added trypsin in cell culture) for cleavage, thus limiting their replication to the respiratory and enteric tracts where appropriate secreted protease is available. In addition, the residue at the +1 position that immediately follows the cleavage site can affect the efficiency of cleavage (i.e., phenylalanine in virulent NDV; leucine in avirulent NDV) [11], [27].

RETRACTED

The cleavage site sequence of APMV-4 (DIQPR↓F) contains a single basic amino acid, present at the -1 position. This resembles the cleavage site sequence of avirulent NDV strains. However, unlike avirulent NDV strains, APMV-4 replicates *in vitro* without added protease and its replication is not augmented by added protease [10]. Interestingly, APMV-4 produces single-cell infections and does not cause syncytium formation that typically is a hallmark of paramyxovirus cytopathic effect (CPE). Thus, the importance of the F protein cleavage site in APMV-4 infectivity and pathogenicity was unclear. To investigate this, we developed a reverse genetics system for APMV-4 and used it to generate 6 APMV-4 mutants whose F protein cleavage sites contained various numbers of basic residues and in some cases were derived directly from paramyxoviruses, including NDV. All the mutants exhibited protease independence, but syncytium formation and enhanced replication *in vitro* were observed only when a furin site was present. However, none of the mutations altered the avirulent nature of APMV-4, as we determined pathogenicity of these viruses using well-established methods for APMV-1, such as mean death time (MDT) in 9-day-old embryonated chicken eggs, intracerebral pathogenicity index (ICPI) in 1-day-old chicks, and using natural route of infection in 2-week-old chickens and in 3-week-old mallard ducks. The parental and mutant viruses replicated better in the natural host ducks than in chickens, but were avirulent in both species. These results suggest that the cleavage site sequence is not the limiting factor for APMV-4 replication and pathogenesis in chickens and ducks.

RETRACTED

## Materials and Methods

### 2.1. Cells and Viruses

The chicken embryo fibroblast cell line (DF1), human epidermoid carcinoma cell line (HEp-2), and African green monkey kidney cell line (Vero) (ATCC, Manassas, VA, USA) were grown in Dulbecco's minimal essential medium (DMEM) with 10% fetal bovine serum (FBS) and maintained in DMEM with 5% FBS. Primary chicken neuronal cells were grown in Neurobasal medium with B-27 supplement (Invitrogen, Carlsbad, CA).

The modified vaccinia virus strain Ankara (MVA) expressing T7 RNA polymerase was kindly provided by Dr. Bernard Moss (NIAID, NIH) and propagated in primary chicken embryo fibroblast cells in DMEM with 2% FBS. APMV-4 strain duck/Hong Kong/D3/75 was obtained from the National Veterinary Services Laboratory (Ames, Iowa). This biologically-derived APMV-4 virus and all of the generated recombinant viruses were grown in the allantoic cavities of 9-day-old specific pathogen free (SPF) embryonated chicken eggs. Virus stocks were quantified by plaque titration on DF1 cells [10] and by hemagglutination (HA) assay with chicken erythrocytes. All experiments involving experimental animals were approved by the committee of IACUC, University of Maryland (protocol number R-09-81) and conducted following the guidelines. All animal care and handling, including euthanasia were conducted according to the procedures of Animal Care and Use committee at the University of Maryland, College Park and guideline of the American Veterinary Medical Association. All efforts were made to minimize discomfort and pain. The personnel conducting this experiment examined infected birds three times a day for clinical symptoms following the well-established scoring system. Birds that show a total score of 0 were considered “normal” while birds showing scores of 1 to 8 were considered “sick.” If a bird presents a score of 2 or 3 in any of the categories above, we increased the monitoring frequency to 3 times daily. Supportive care was provided (soft food) for animals that show scores of 2 or 3. If the condition worsens or does not improve after it has reached a score of 3, it was euthanized as it is considered that the bird has reached a moribund state. If necessary, Dr. Yanjin Zhang, facility veterinarian in the department was contacted to determine whether the bird needs to be euthanized or requires supportive care. Supportive care (soft food, subcutaneous fluids) was provided if it does not interfere with the objective of this study. Birds were anesthetized and killed by an overdose of isoflurane, the inhalant anesthetic. Briefly, sterile cotton gauze was placed in the bottom of a sterile bell jar and was covered with a wire mesh. Approximately, 1 to 2 ml of isoflurane was added into the cotton gauze. The bird was placed in the jar and the lid was closed quickly. The bird was removed from the jar after cessation of breathing.

RETRACTED

### 2.2. Construction of Plasmid Bearing the Full-Length Antigenomic cDNA of APMV type 4 and Support Plasmids

A full-length antigenomic cDNA of APMV-4 was constructed based on the complete consensus sequence of APMV-4 strain duck/Hong Kong/D3/75 (GenBank accession no. FJ177514). Based on this sequence, gene-specific primers were designed for RT-PCR using as template RNA from APMV-4 virions. Six fragments were generated and were inserted into a modified pBR322 [6] using five restriction sites (SbfI, SnaBI, MluI, NotI, and PvuI) that were introduced into untranslated regions (UTRs) (Fig. 1). Fragments bearing the N, P, M, F, HN, and L genes were consecutively inserted into pBR322. To construct support plasmids, cDNA fragments containing the ORFs of the N, P, and L genes of APMV-4 were generated by RT-PCR. The N and P ORFs were cloned individually into plasmid pTM-1 between NcoI and XhoI sites. The L gene ORF was cloned into plasmid pGEM between AatII and SacI sites by a two-step cloning procedure using XmaI site as the third restriction site. The full-length cDNA of APMV-4 in pBR322, the N and P ORFs in pTM-1, and the L ORF in pGEM were sequenced in their entirety.

**Figure 1:** Construction of a cDNA clone encoding a full-length antigenomic RNA of APMV-4, and the introduction of modified F genes. The APMV-4 cDNA was assembled between the T7 promoter (to the left) and the hepatitis delta virus antigenomic ribozyme sequence followed by a T7 RNA polymerase transcription-termination signal (to the right). Assembly of the cDNA employed SbfI, SnaBI, MluI, NotI, and PvuII sites that were introduced into untranslated regions. To generate F protein cleavage site mutant viruses, the cDNA fragment containing the F gene was swapped using the MluI and NotI sites.

Infectious APMV-4 was generated as previously described for NDV [6]. Briefly, HEp-2 cells were transfected with three plasmids individually encoding the N, P, and L proteins (2.0 µg, 1.0 µg, and 0.5 µg per single well of a six-well dish, respectively) and a fourth plasmid encoding the full-length antigenome (5.0 µg) using Lipofectamine (Invitrogen) and simultaneously infected with vaccinia MVA expressing T7 RNA polymerase at a multiplicity of infection (MOI) of 1 PFU/cell. Two days after transfection, supernatant was inoculated into the allantoic cavity of 9-day-old embryonated chicken eggs. Recovery of the virus was confirmed by hemagglutination assay using 1% chicken red blood cells (RBCs). The presence of unique restriction enzyme sites in the recovered virus was confirmed by RT-PCR analysis.

RETRACTED

### 2.3. Generation of rAPMV-4 with Mutations at Cleavage Site Sequence of the F Protein

Initially, the wild-type APMV-4 F protein cleavage site (DIQPR↓F) was changed to the naturally occurring cleavage sites of mesogenic NDV strain Beaudette C (BC) (RRQKR↓F), APMV-3 (RPRGR↓L), and APMV-5 (KRKKR↓F). Mutagenesis was performed by overlapping PCR on the MluI-NotI fragment bearing the F gene (Fig. 1), which was then cloned into the full-length antigenomic APMV-4 cDNA. Sequence analysis confirmed the absence of adventitious mutations in the MluI-NotI fragment. Transfection for virus recovery was conducted as described above. We readily recovered the mutant bearing the NDV BC cleavage site (rAPMV-4/Fc BC) but failed to recover the other two mutants in five separate transfection experiments in which the wild type rAPMV-4 virus was readily recovered each time. We noted that the F protein cleavage site sequence of APMV-4 has a glutamine residue at the -3 position, and we previously had observed that the glutamine residue at the -3 position in the cleavage site of NDV is important in virus replication and pathogenicity [28]. Therefore, we replaced the arginine and lysine residues at the -3 position in the cleavage site sequences of APMV-3 and APMV-5, respectively, with glutamine to yield the cleavage sites RPQGR↓F and KRQKR↓F, respectively, which were then introduced into rAPMV-4 (Table 1). We also prepared rAPMV-4 mutants containing the cleavage site from the avirulent NDV strain LaSota (GRQGR↓L), Sendai virus (SV) (VPQSR↓F), and human parainfluenza virus type 1 (PIV1) (NPQTR↓F) (Table 1). These manipulations involved the MluI-NotI fragment noted above, and sequence analysis confirmed the absence of adventitious mutations in each mutated fragment. Each of these mutant viruses was readily recovered, and the sequences of the F protein cleavage sites were confirmed by RT-PCR analysis of recovered virus.

**Table 1:** Cleavage site sequence of parental and recombinant APMV-4 viruses and pathogenicity in MDT and ICPI assays.

Virus	Cleavage site		MDT^a^	ICPI^b^
	Sequence	Furin motif		
wtAPMV-4	DIQPR ↓F	-	>168	0.00
rAPMV-4	DIQPR ↓F	-	>168	0.00
rAPMV-4/Fc type 3-Q	RPQGR↓F	-	>168	0.00
rAPMV-4/Fc type 5-Q	KRQKR↓F	+	>168	0.00
rAMPV-4/Fc BC	RRQKR↓F	+	>168	0.00
rAMPV-4/Fc LaSota	GRQGR ↓L	-	>168	0.00
rAMPV-4/Fc SV	VPQSR↓F	-	>168	0.00
rAMPV-4/Fc PIV 1	NPQTR↓F	-	>168	0.00

a Mean embryo death time (MDT): the mean time (h) for the minimum lethal dose of virus to kill all of the inoculated embryos. Pathotype definition: virulent strains, <60 h; intermediate virulent strains, 60 to 90 h; avirulent strains, >90 h.

b Intracerebral pathogenicity index (ICPI): pathogenicity of NDV in 1-day-old SPF chicks following intracerebral inoculation. Pathotype definition: virulent strains, 1.5–2.0; intermediate virulent strains, 0.7–1.5; and avirulent strains, 0.0–0.7.

RETRACTED

### 2.4. Expression and Cleavage Efficiency of the F Protein

Incorporation of wild-type and mutated F proteins into the virions was analyzed by Western blot using an antiserum raised against a synthetic peptide from the F protein of APMV-4. The parental and APMV-4 mutant viruses were grown in embryonated eggs and subjected to discontinuous sucrose gradients to obtain partially purified stocks [29]. In addition, cleavage efficiency of wild-type and mutated F proteins were evaluated in virus-infected DF1 cells at an MOI of 0.1, and cell lysates collected at 24 h post-infection (hpi) were subjected to Western blot analysis with anti-APMV-4 F rabbit polyclonal antiserum [13], [30]. Surface expression of the F protein was evaluated on virus-infected DF1 cells at an MOI of 0.1. At 24 h post-infection (hpi), the cells were labeled with the anti-peptide antiserum against the F protein of APMV-4 followed by anti-Alexa Fluor 488 antibody, fixed with 4% paraformaldehyde, and analyzed by flow cytometry (AriaII, BD Bioscience) with Flowjo program (Tree Star, Inc.).

### 2.5. Growth Characteristics of Parental and Cleavage site Mutant APMV-4 Viruses in DF1 Cells

The growth characteristics of the parental and recombinant viruses were evaluated in DF1 and Vero cells. The plaques were fixed and immunostained using a previously-described antiserum raised against gel-purified N protein of partially-purified APMV-4 virions [31]. The requirement for supplementation of exogenous protease for cleavage of the F protein was determined by addition of either 1 µg/ml of acetyl trypsin or 5% chicken egg allantoic fluid [32] in preliminary experiments. Protease supplementation was not used in subsequent experiments. The growth kinetics of parent and mutant viruses was evaluated in DF1 cells at a multiplicity of infection (MOI) of 1 or 0.01 [33]. Virus titers in the collected supernatants were quantified in DF1 cells by limiting dilution and immunostaining with N-specific antiserum and expressed as 50% tissue culture infectious dose (TCID_50_/ml) by the end-point method of Reed and Muench [34].

RETRACTED

### 2.6. Mean Death Time and Intracerebral Pathogenicity Index Tests

The pathogenicity of parental and mutant APMV-4 viruses was determined by the mean death time (MDT) test in 9-day-old SPF embryonated chicken eggs and by the intracerebral pathogenicity index (ICPI) test in 1-day-old SPF chicks [35]. Briefly, for the MDT test, a series of 10-fold dilutions of infected allantoic fluid (0.1 ml) was inoculated into the allantoic cavities of five 9-day-old eggs per dilution and incubated at 37°C. The eggs were examined once every 8 h for 7 days, and the time of embryo death was recorded. The MDT was determined as mean time (h) for the minimum lethal dose of virus to kill all the inoculated embryos. The criteria for classifying the virulence of NDV isolates are: <60 h, virulent strains; 60 to 90 h, intermediate virulent strains; and >90 h, avirulent strains. For the ICPI test, 0.05 ml of a 1∶10 dilution of fresh infective allantoic fluid for each virus was inoculated into group of 10 1-day-old SPF chicks via the intracerebral route. At each observation, the birds were scored as follows: 0 if normal; 1 if sick; and 2 if dead. The ICPI is the mean of the score per bird per observation over the 8-day period. Highly virulent velogenic viruses give values approaching 2, and avirulent or lentogenic strains give values at or close to 0.

### 2.7. Neurotropism of Parental and Cleavage Site Mutant APMV-4 Viruses

To evaluate neurotropism of parental and mutant APMV-4 *in vitro*, primary chicken neuronal cells were prepared from 9-day-old chicken embryos for virus infection [27], [36]. After 72 h of infection, the cells were fixed with 4% paraformaldehyde, permeabilized with 0.2% Triton, stained with antiserum against the N protein and polyclonal antibodies against a neuronal marker (anti-neuron specific beta III tubulin antibody, abcam®, Cambridge, MA) followed by anti-Alexa Fluor 488 and 594 antibodies, and then analyzed by confocal microscopy. In addition, during the infection period, virus titers in the collected supernatants at 12-h intervals were quantified in DF1 cells by immunostaining with N-specific antiserum as described above.

To determine the ability of parental and mutant viruses to replicate in chicken brains, 1-day-old SPF chicks in groups of ten were inoculated with 0.05 ml of a 1∶10 dilution of fresh infective allantoic fluid for each virus via the intracerebral route. Two birds per group were sacrificed daily until 5 days post-infection (dpi) and analyzed for infectious virus by immunostaining with N-specific antiserum in DF1 cells.

RETRACTED

### 2.8. Replication of Parental and Mutant APMV-4 Viruses in Chickens and Ducks Following Inoculation of the Respiratory Tract

Replication was evaluated in 1-day-old chicks, 2-week-old chickens, and 3-week-old mallard ducks following respiratory tract inoculation. One-day-old chicks in groups of 8 were inoculated with 100 µl of each virus (256 HA units/bird) via the intranasal route. At 3 dpi, one half of the chicks from each group were sacrificed and tissue samples (lung, trachea, spleen, and brain) were collected for virus titration by limiting dilution and immunoperoxidase assay. The remaining three chicks per group were observed daily for 14 days for any clinical signs and then sacrificed for virus titration of various tissues as described above. Sera were collected from the chicks on 14 dpi and evaluated for seroconversion by HI assay [35]. Two-week-old SPF chickens in groups of six were inoculated with 200 µl of each virus (256 HA units/bird) by the intranasal route. Three birds from each group were sacrificed at 4 dpi and tissues samples (lung, trachea, spleen, and brain) were collected for virus titration. Virus titers in DF1 cells were determined by limiting dilution and immunostaining as described above. To obtain more sensitive detection of replication, tissue samples from the 2-week-old chickens also were inoculated into 9-day-old embryonated chicken eggs [36]. At 3 dpi, the allantoic fluids were tested for virus growth by HA assay. The remaining three birds per group were observed daily for 14 days for any clinical signs and then sacrificed for virus titration of various tissues as described above. Sera were collected from the chickens on 14 dpi and evaluated for seroconversion by HI assay [35]. Three-week-old mallard ducks in groups of six were infected with 500 µl of each virus (256 HA units/bird) via the combined intranasal and intratracheal routes. For virus titrations, three ducks per group were sacrificed at 4 dpi and used for collection of tissue samples (lung, trachea, spleen, and brain). The remaining ducks were observed daily for 10 days for any clinical signs.

### 2.9. Histopathology and Immunohistochemistry

The various tissue samples harvested from infected 2-week-old chickens and 3-week-old ducks were fixed in phosphate-buffered formalin (10%), embedded in paraffin, and sectioned (Histoserv, Inc., Germantown, MD). Sections from mock-infected birds were used as controls. The tissues were deparaffinized, rehydrated, and subsequently, immunostained to detect viral N protein [36].

## Results

### 3.1. Development of an APMV-4 Reverse Genetics System

A cDNA clone of the antigenomic RNA of APMV-4 was constructed from six cDNA segments that were synthesized by RT-PCR from virion-derived genomic RNA (Fig. 1). The cDNA segments were cloned in a sequential manner into the low-copy-number plasmid pBR322/dr [6] between a T7 promoter (TAATACGACTCACTATAGG) and the hepatitis delta virus ribozyme sequence. The resulting APMV-4 cDNA in the plasmid pBR322/dr/APMV-4 is a faithful copy of the published consensus sequence for the APMV-4 antigenome [10] except for 10 silent nucleotide changes that were introduced to create five new unique restriction enzyme sites used in the construction (SbfI, SnaBI, MluI, NotI, and PvuI, Fig. 1). This construct contains a T7 promoter that initiates the encoded antigenomic RNA with three extra G residues at its 5′ end, which was previously shown for NDV to increase the efficiency of T7 polymerase transcription without interference with viral recovery [6]. Three support plasmids were constructed that express the N, P, and L ORFs of APMV-4 under the control of the T7 promoter. Recombinant APMV-4 (rAPMV-4) was readily recovered by transfection of the antigenome plasmid into HEp-2 cells together with plasmids encoding the N, P, and L proteins, necessary for viral RNA replication and transcription. Recovery of the virus was facilitated by inoculating the transfection mixture into 9-day-old embryonated chicken eggs, since APMV-4 replicates to high titer in embryonated chicken eggs than in cell culture. Furthermore, the recombinant virus did not require exogenous protease during transfection and passage, which is consistent with the previous observation that replication of biologically-derived wild-type APMV-4 is unaffected by added protease [10].

RETRACTED

### 3.2. Generation of Cleavage Site Mutant APMV-4 Viruses

The F protein cleavage site of APMV-4 has a single basic amino acid residue (DIQPR↓F), and thus lacks the preferred cleavage site for the protease furin (RX[K/R]R↓). Initially, we constructed and attempted to recover three mutant rAPMV-4 viruses bearing the naturally occurring F protein cleavage sites of three different viruses: namely, the neurovirulent NDV strain BC (RRQKR↓F), which contains four basic amino acids as well as the furin motif; APMV-3 (RPRGR↓L), which has three arginine residues but lacks the furin motif; and APMV-5 (KRKKR↓F), which has five tandem basic residue and contains the furin motif [13]. Somewhat surprisingly, virus recovery was successful only with the mutant containing the cleavage site sequence of NDV BC (rAPMV-4/Fc BC, Table 1); the other two mutants could not be recovered in five different attempts in which positive controls were readily recovered.

We had previously found that the presence of a glutamine residue at the -3 position in the cleavage site of NDV is important in virus replication and pathogenicity [28]. We also noted that the F protein cleavage site sequence of unmodified APMV-4 has glutamine residue at the -3 position. Glutamine also is present at position -3 in the NDV BC F cleavage site, but not in the cleavage sites of APMV-3 or -5. Therefore, we modified these latter two sites to contain a glutamine at position -3 (RPQGR↓F and KRQKR↓F, respectively) and inserted these sites into rAPMV-4. Virus was readily recovered from these cDNAs (rAPMV-4/Fc type 3-Q and rAPMV-4/Fc type 5-Q, respectively, Table 1), suggesting an important role for glutamine at position -3 in F protein function and virus recovery. We also prepared rAPMV-4 mutants bearing the naturally-occurring F cleavage site sequences of three other viruses: namely, avirulent NDV strain LaSota (GRQGR↓L), SV (VPQSR↓F), and human PIV-1 (NPQTR↓F). Each of these contained a glutamine residue in the -3 position. Each of these additional mutants was readily recovered (yielding viruses rAPMV-4/Fc LaSota, rAPMV-4/Fc SV, and rAPMV-4/Fc PIV1, Table 1). Added protease was not necessary for any of these recoveries. To evaluate genetic stability, the viruses were passaged five times in 9-day-old embryonated chicken eggs, and the sequence of the F gene was confirmed, showing that the introduced mutations were maintained without any adventitious mutations. Out of the six mutant viruses that were successfully recovered, only two had furin motifs in the F protein cleavage site: namely, rAPMV-4/Fc BC and rAPMV-4/Fc type 5 Q (Table 1)

The viral proteins in partially purified parental and chimeric viruses were analyzed by Western blot using antiserum raised against a synthetic peptide representing amino acids 358 to 372 of the APMV-4 F protein. The protein composition of the wild-type and recombinant viruses was verified by Coomassie blue staining of the purified viral proteins (Fig. 2A). This confirmed that all of the recombinant viruses contained a similar pattern of the major structural proteins, suggesting that the various mutations of the F protein cleavage site did not affect virion assembly (Fig. 2B).

RETRACTED

**Figure 2:** Analysis of proteins present in virions of parental and F protein cleavage site mutant APMV-4 viruses, and cell-surface expression of the viral F protein. (A) Virus that was partially purified from infected chicken egg allantoic fluids by sucrose step gradients was separated by electrophoresis, and the gel was stained with Coomassie brilliant blue. Lanes: 1. Biologically-derived APMV-4, 2. rAPMV-4, 3. rAPMV-4/Fc type 3-Q, 4. rAPMV-4/Fc type 5-Q, 5. rAMPV-4/Fc BC, 6. rAMPV-4/Fc Las, 7. rAMPV-4/Fc SV, and 8. rAMPV-4/Fc PIV-1 (B) Incorporation of wild-type and mutated F proteins into the virions was further analyzed by Western blot. The separated proteins in the gel (8%) under reducing condition (in panel A) were transferred into a membrane, and the F protein was detected by using an antiserum raised against a synthetic peptide from the F protein of APMV-4. (C) Surface expression of the F protein on infected DF1 cells. DF1 cells were infected with each virus (MOI of 0.1) and, at 24 h post-infection, were stained with anti-peptide antiserum against the F protein followed by anti-Alexa Fluor 488 antibody, and were analyzed by flow cytometry.

The effect of the cleavage site mutations on the surface expression of the F protein in DF1 cells was further evaluated by flow cytometry analysis. This showed that wild type biologically-derived APMV and its recombinant version rAPMV-4 were indistinguishable with regard to the level of surface expression of the F protein (Fig. 2C). Most of mutant viruses also had similar levels of surface expression to those of the biological and recombinant parental viruses. There was one exception: the level of expression of F protein by the rAPMV-4/Fc BC virus was 275% that of the parental viruses, indicating that expression was substantially increased by introduction of the NDV BC cleavage site.

### 3.3. Cytopathic Effect and Growth Characteristics of APMV-4 Mutant Viruses in Vero and DF1 Cells

We previously reported that biologically-derived wild-type APMV-4 replicates in Vero and DF1 cells without supplementation by exogenous protease, and causes single-cell infections in cell culture, with cell rounding and detachment but without the formation of syncytia. Furthermore, replication and syncytium formation were not enhanced by the addition of protease [10]. To investigate the effects of the mutant cleavage site sequences on syncytium formation by APMV-4, DF1 cells were infected with the parental biologically-derived wild-type APMV-4, its recombinant version rAPMV-4, and the six different mutant viruses. The cells were visualized 72 hpi by photomicroscopy directly (Fig. 3A) and following immunostaining with antiserum against the APMV-4 N protein (Fig. 3B). In parallel, the ability of the viruses to produce plaques was tested on DF1 cells under 0.8% methylcellulose overlay (not shown). Biologically-derived and recombinant wild-type APMV-4 produced similar CPE (i.e., single-cell infections) in DF1 cells (Fig. 3). The two viruses did not produce plaques under methylcellulose overlay in the presence or absence of exogenous protease (i.e., acetyl trypsin or chicken egg allantoic fluid, data not shown) up to 72 hpi. Among the F protein cleavage site mutant viruses, only rAPMV-4/Fc BC produced distinctive syncytia (Fig. 3) and plaques (not shown) that resembled those of NDV strain BC. rAPMV-4/Fc type 5-Q showed sporadic syncytium formation both in DF1 cells, but failed to produce distinguishable plaques. In contrast, the other four mutant viruses produced CPE that was characterized by single-cell infections, cell rounding, and detachment of virus-infected cells, similar to that of the wild-type APMV-4 parents, indicating that these mutations in the F protein cleavage site did not affect viral CPE. Furthermore, the addition of acetyl trypsin or chicken egg allantoic fluid to the cell cultures as a source of exogenous protease did not result in increased virus replication, syncytium, and plaque formation for any virus (data not shown). The two APMV-4 mutants that were able to produce syncytia in cell culture, rAPMV-4/Fc BC and rAPMV-4/Fc type 5-Q, were also the two that contained a furin motif in the F protein cleavage site. Western blot analysis showed that the F protein of these two mutants was efficiently cleaved in DF1 cells, whereas other mutants that did not produce syncytia showed incomplete cleavage of F protein (Fig. 3C). Our results suggest that efficient cleavage of APMV-4 F protein is required for syncytium formation. Supplementation of 10% allantoic fluid did not change the status of wt and mutant F proteins (data not shown).

RETRACTED

**Figure 3:** Production of cytopathic effect and proteolytic cleavage of the F0 proteins of parental and F protein cleavage site mutant APMV-4 viruses. (A) DF1 cells in six-well plates were infected with the indicated viruses at a multiplicity of infection (MOI) of 0.1 PFU/cell and incubated for 72 h. (B) The viral plaques in the infected cells were visualized by immunoperoxidase staining using antiserum against the N protein of APMV-4; viral antigen is stained red. (C) Proteolytic cleavage of the F0 proteins of parental and mutant viruses in infected DF1 cells was analyzed by Western blot (I) in triplicate. The positions of the precursor protein F0 and the cleavage product F1 are indicated. The relative levels of the F0 and F1 proteins in the Western blot images were measured by Bio-Rad Gel Image analysis, and the efficiency of cleavage was determined by dividing the amount of F1 by the amount of F1 plus F0 (II).

We evaluated the replication kinetics of parental and F protein cleavage site mutant viruses in DF1 cells (Fig. 4). In one experiment, cells were infected at a low MOI of 0.01 in order to evaluate multi-cycle replication. Biological wild-type APMV-4 and its recombinant version rAPMV-4 did not exhibit efficient multi-cycle replication in DF1 cells, yielding very low titers (<10^2^ TCID_50_/ml, Fig. 4A). However, two of the mutant viruses exhibited substantial increases in the kinetics and magnitude of replication. rAPMV-4/Fc BC grew much better than any other APMV-4 mutants, reaching a maximum titer of 5.0×10^5^ TCID_50_/ml at 84 hpi. rAPMV-4/Fc type 5-Q also replicated substantially better than other mutant viruses, reaching a maximum titer of 10^2^ TCID_50_/ml at 84 hpi. Efficient replication of the other four APMV-4 mutant viruses was not detected, which is similar to that of the biological and recombinant wild-type viruses (<10^2^ TCID_50_/ml). We further evaluated virus replication in DF1 cells by infecting at an MOI of 1. Under these conditions, biologically-derived wild-type APMV-4 and its recombinant version rAPMV-4 reached a maximum titer of 10^3^ TCID_50_/ml at 72 hpi. Among the mutant viruses, rAPMV-4/Fc BC and rAPMV-4/Fc type 5-Q grew to titers of 5.0×10^5^ TCID_50_/ml at 24 hpi and 8.0×10^4^ TCID_50_/ml at 72 hpi, respectively, thus replicating to a 100-fold higher titer compared to the parental viruses. The other four mutant viruses replicated to maximum titers similar to those of the parental viruses. The increased *in vitro* replication of rAPMV-4/Fc BC and rAPMV-4/Fc type 5-Q (Fig. 4) correlated with the ability to form syncytia (Fig. 3), enhanced surface expression of the F protein (Fig. 2C), and the presence of a furin motif (Table 1). On the contrary, APMV-4 wild-type and mutant viruses grew to high titer (2^8^ HAU/ml) in embryonated eggs, indicating that probably, there is a protease in the cells of allantoic membrane that efficiently cleaves the F protein of APMV-4.

RETRACTED

**Figure 4:** Replication of parental and F protein cleavage site mutant APMV-4 viruses in DF1 cells. The growth kinetics of parental and recombinant APMV-4 viruses was determined by infecting DF1 cells with each virus at an MOI of 0.01 (A) and 1 (B). The viral titers were determined by limiting dilution on DF1 cells and immunostaining with antiserum raised against the N protein of APMV-4.

### 3.4. Evaluation of the Pathogenicity of Wild-Type and Cleavage Site Mutant APMV-4 Viruses in Chickens by the MDT and ICPI Tests

The pathogenicity of the wild-type and mutant APMV-4 viruses was evaluated by the standard, internationally-accepted pathogenicity tests for NDV, namely the MDT assay in embryonated chicken eggs and the ICPI assay in 1-day-old chicks (Table 1). Biologically-derived wild-type APMV-4 and its recombinant version rAPMV-4 were identical with regard to the values of MDT and ICPI, which were >168 h and 0.00, respectively, indicating their avirulence in chickens. Interestingly, the MDT and ICPI values of each of the six mutant viruses were identical to those of the parental APMV-4 viruses. None of the viruses caused the death of any of the chicken embryos within the standard 7-day time limit for assay. Chicks infected with each mutant virus had no apparent clinical signs during the 8-day period of the ICPI test. Thus, all of the APMV-4 viruses in this study were highly attenuated, and none of the various mutations in the cleavage site of the F protein had any discernable effect on the virulence of APMV-4.

RETRACTED

### 3.5. Replication of Parental and Mutant APMV-4 in Neuronal Cells *in vitro* and in the Brains of 1-day-old Chicks

To evaluate possible neurotropism of the parental and mutant APMV-4 viruses, we assayed their ability to replicate in primary chicken neuronal cells *in vitro*. First, neuronal cell cultures were infected with the panel of viruses at an MOI of 0.1 PFU. The cells were fixed at 72 hpi, immunostained with antiserum against the N protein of APMV-4, and visualized by confocal microscopy (Fig. 5). Neurovirulent NDV strain BC was used as a control, and the expression of N protein by this virus was clearly detected in dendrites and axons. In contrast, N protein expression could not be detected in the case of biologically-derived wild-type APMV-4 or its recombinant version. Among the F protein cleavage site mutant viruses, N protein expression was detected sporadically in the case of rAPMV-4/Fc BC, but was not detected with any other mutant. We also examined replication in the neuronal cell cultures by collecting supernatants from the cultures at 12 h intervals and assaying for infectious virus by titration in DF1 cells (not shown). Although neurovirulent NDV strain BC was able to grow to 5.5 TCID_50_/ml at 72 hpi, none of the parental or mutant APMV-4 viruses, including rAPMV-4/Fc BC, were detected, indicating their inability to replicate in these cultures of primary chicken neuronal cells (data not shown).

**Figure 5:** Replication of parental and F protein cleavage site mutant APMV-4 viruses in primary chicken neuronal cells. Neuronal cells were infected with APMVs at an MOI of 0.1. At 48 hpi, the cells were fixed with 4% paraformaldehyde, permeabilized with 0.2% Triton X-100, stained with a neuronal marker (anti-neuron specific beta III tubulin polyclonal antibodies) and antiserum against the N protein of APMV-4 followed by anti-Alexa Fluor 488 and 596, and then analyzed by confocal microscopy. The neuronal marker and viral N protein stained red and green, respectively.

We investigated the ability of the parental and mutant viruses to replicate in chicken brains by inoculating 1-day-old chicks via the intracerebral route. The infected chickens were sacrificed daily and brain tissue was collected for virus titration (Fig. 6). We included neurovirulent NDV strain BC and avirulent NDV strain LaSota as controls. In chicks infected with NDV strain BC, virus replication reached a peak titer of >6.0 log_10_ TCID_50_/g at 2 dpi, and all of the infected chicks died on 3 dpi. The LaSota strain was detected at low titer on day 1, but was not detected on subsequent days and did not cause disease or death during the 5 days of observation. Replication of the parental and mutant APMV-4 viruses was not detectable on any day, and there was no detectable disease or death, indicating that wild type APMV-4 does not replicate detectably in chicken brains, and that none of the cleavage site mutations gained this ability.

RETRACTED

**Figure 6:** Growth kinetics of parental and F protein cleavage site mutant APMV-4 viruses in the brains of 1-day-old chicks. Ten 1-day-old SPF chicks were inoculated with the indicated parental or mutant viruses via the intracerebral route. Two birds in each group were sacrificed daily until 5 dpi. Brain tissue samples were harvested and virus titers were determined by limiting dilution in DF1 cells and immunostaining with antiserum against the N protein of APMV-4. Each bar represents mean and standard error of the mean of duplicate samples.

### 3.6. Replication of Parental and Mutant APMV-4 Viruses in 1-day-old and 2-week-old Chickens

We next evaluated replication and tissue tropism of the parental and mutant APMV-4 viruses in 1-day-old and 2-week-old chickens following intranasal inoculation. One-day-old chicks were infected, and one half of each group was sacrificed at 3 dpi and tissue samples (trachea, lung, spleen, and brain) were collected for virus titration by limiting dilution. Replication of parental and mutant APMV-4 in 1-day-old chicks was detected only in the trachea, with titers that were low and ranged from 1.5 to 2.2 log_10_ TCID_50_/g (data not shown). The viruses were not detected in other collected tissue samples (data not shown). The remaining birds in each group were observed daily for a total of 14 days for any clinical signs and then sacrificed for virus titration of various tissues as described above. Virus was not detected in any of the 14 dpi samples (data not shown). Clinical signs of illness were not observed in any of the infected groups.

Two-week old chickens were inoculated by the intranasal route with the various viruses, and one half of the birds in each group were sacrificed at 4 dpi and tissue samples (trachea, lungs, spleen, and brain) were collected for virus titration by limiting dilution. Replication of parental and mutant APMV-4 was not detected in any the harvested tissue samples from 4 dpi (data not shown). Since APMV-4 does not replicate efficiently in cell culture (Fig. 4), but replicates efficiently in embryonated eggs, the tissue homogenates from the experiment with the 2-week-old birds also were inoculated into eggs to as a more sensitive assay to detect possible in the various tissues. For the samples from 4 dpi, replication of parental and mutant APMV-4 viruses were detected sporadically (in 1 out of 3 birds in each case) in the trachea from chickens infected with biologically-derived wild-type APMV-4, rAPMV-4/Fc type 5-Q, rAMPV-4/Fc BC, rAMPV-4/Fc LaSota, and rAMPV-4/Fc SV (Table 2). Virus was not detected in samples from chickens infected with rAPMV-4, rAPMV-4/Fc type 3-Q, or rAPMV-4/Fc PIV1. This sporadic pattern indicated that replication in 2-week-old chickens was not significantly different between the parental and the various mutant APMV-4 viruses. The remaining birds in each group were observed daily for a total of 14 days for any clinical signs and then sacrificed for virus titration of various tissues by limiting dilution and by inoculation of embyonated eggs as described above. Virus was not detected in any of the 14 dpi samples (data not shown). Clinical signs of illness were not observed in any of the infected groups.

RETRACTED

**Table 2:** Replication of parental and F protein cleavage site mutant APMV-4 viruses in 2-week-old chickens.

Virus	Virus replication in embryonated eggs^a^			
	Brain	Trachea	Lung	Spleen
wtAPMV-4	0/3	1/3	0/3	0/3
rAPMV-4	0/3	0/3	0/3	0/3
rAPMV-4/Fc type 3-Q	0/3	0/3	0/3	0/3
rAPMV-4/Fc type 5-Q	0/3	1/3	0/3	0/3
rAMPV-4/Fc BC	0/3	1/3	0/3	0/3
rAMPV-4/Fc LaSota	0/3	1/3	0/3	0/3
rAMPV-4/Fc SV	0/3	1/3	0/3	0/3
rAMPV-4/Fc PIV 1	0/3	0/3	0/3	0/3

a Groups of 2-week-old chickens were inoculated with each virus by the intranasal route. Three birds from each group were sacrificed, and tissues samples (brain, trachea, lung, and spleen) were collected and homogenized. To investigate virus replication, aliquots (100 µl each) of the collected samples on 4 dpi was inoculated into three eggs, and allantoic fluids were collected on 3 dpi. Virus replication was determined by hemagglutination assay.

Tissue samples collected on 4 dpi from the 2-week-old chickens also were evaluated for histopatholgy (data not shown). This revealed similar microscopic findings for the parental and cleavage site mutant viruses. Specifically, the trachea infected with parental and all of the mutant APMV-4 viruses except for rAPMV-4/Fc BC exhibited minimal lymphocytic tracheitis and mild multifocal mucosal attenuation, whereas the trachea infected with rAPMV-4/Fc BC showed mild lymphocytic tracheitis and mild to moderate multifocal mucosal attenuation (data not shown). In general, lung sections exhibited mild to moderate, multifocal, lymphocytic to lymphohistiocytic bronchitis with minimal perivascular and parabronchial interstitial inflammation. Significant lesions were not found in any of the brain or spleen tissues. These results suggested that parental and cleavage site mutant APMV-4 viruses were avirulent in chickens, and their replication was mostly restricted to the trachea.

RETRACTED

Virus replication in 1-day-old and 2-week-old chickens infected with parental and mutant APMV-4 viruses was further investigated by measuring seroconversion at 14 dpi in the studies described above (Fig. 7). Sera were analyzed by HI assay using chicken erythrocytes. All of the infected chickens from each age group seroconverted at 14 dpi. Although parental and mutant APMV-4 viruses replicated with low systemic spread, all viruses were able to induce a good humoral immune response. In general, sera collected from chickens infected as 1-day-old chicks showed higher HI titers than those infected as 2-week-old-chickens. Also, certain mutant viruses, such as rAMPV-4/Fc BC and rAMPV-4/Fc SV, induced slightly better immune response than did parental APMV-4.

**Figure 7:** Induction of serum antibodies in response to infection of 1-day-old and 2-week-old chickens with parental and F protein cleavage site mutant APMV-4 viruses. Chickens were inoculated with each virus (256 HA units) by the intranasal route in the same experiment as Table 2. Sera were collected at 14 dpi and evaluated for virus-specific antibodies by a hemagglutination inhibition assay using chicken erythrocytes.

### 3.7. Replication of APMV-4 Parental and Mutant Viruses in 3-week-old Ducks

Since biologically-derived wild-type APMV-4 was isolated originally from a mallard duck, we evaluated the wild-type and mutant APMV-4 viruses in this species. Three-week-old ducks (six each) were inoculated by the combined intranasal and intratracheal routes with the various APMV-4 viruses. One half of each group was sacrificed at 4 dpi and tissue samples (trachea, lungs, spleen, and brain) were collected for virus titration by limiting dilution in DF1 cells. Replication of parental and mutant APMV-4 viruses was not detected by this assay in any of the tissue samples (data not shown). However, using the more sensitive assay of inoculating tissue homogenates into embryonated eggs, virus was detected in most of the samples of trachea, lungs, and spleens, but not in the brain (Table 3). For example, both biologically-derived wild-type AMPV-4 and its recombinant version rAPMV-4 were detected in the trachea and lung of one or two each out of three ducks in each group, and rAPMV-4 was detected in the spleen of a single duck. All the F protein cleavage site mutant viruses were also detected in the trachea and lungs of one or two ducks per group. Among the mutant viruses, rAMPV-4/Fc type 3-Q, rAMPV-4/Fc BC, and rAMPV-4/Fc SV were each detected in the spleen of a single duck.

RETRACTED

**Table 3:** Replication of parental and F protein cleavage site mutant APMV-4 viruses in 3-week-old ducks.

Virus	Virus replication in embryonated eggs^a^			
	Brain	Trachea	Lung	Spleen
wtAPMV-4	0/3	2/3	1/3	0/3
rAPMV-4	0/3	1/3	1/3	1/3
rAPMV-4/Fc type 3-Q	0/3	2/3	1/3	1/3
rAPMV-4/Fc type 5-Q	0/3	2/3	1/3	0/3
rAMPV-4/Fc BC	0/3	2/3	2/3	1/3
rAMPV-4/Fc LaSota	0/3	2/3	2/3	0/3
rAMPV-4/Fc SV	0/3	2/3	2/3	1/3
rAMPV-4/Fc PIV 1	0/3	1/3	1/3	0/3

a Groups of 3-week-old ducks were inoculated with each virus by the combined intranasal and intratracheal routes. Three birds from each group were sacrificed, and tissues samples (brain, trachea, lung, and spleen) were collected on 4 dpi and homogenized. To confirm the virus replication, aliquots (100 µl each) of the collected samples were inoculated into three eggs, and allantoic fluids were collected on 3 dpi. Virus replication was determined by hemagglutination assay.

Histopathological examinations of tissue samples collected on 4 dpi also showed similar patterns between parental and mutant viruses (Fig. 8A). In the trachea, there was mild to moderate lymphocytic tracheitis with mild to moderate multifocal mucosal attenuation and reduction of tracheal mucous glands. Lung sections exhibited moderate to marked multifocal, lymphohistiocytic bronchointerstitial pneumonia with moderate perivascular cuffing in the pulmonary interstitium. Spleen sections showed moderate reactive lymphoid hyperplasia characterized by expansion of the white pulp by reactive lymphocytes and increased size and cell density of lymphoid follicles. However, microscopic lesions were not found in the brain tissues. The presence of viral antigens in various tissues was investigated by immunohistochemistry analysis. Deparaffinized sections of the virus-infected and uninfected control tissue were immunostained using antiserum against the N protein of APMV-4. Viral antigens were detected in tissue samples that were also positive by virus isolation, confirming that the detection of virus in harvested tissue indeed was associated with infection of the organ. This is illustrated with representative virus, rAPMV-4, in Fig. 8B. In the trachea, the presence of antigens for most APMV-4 was detected in the epithelial lining of trachea. In the lungs, viral antigens were mostly localized in the epithelium surrounding the medium and small bronchi. Sporadic distribution of viral antigens was found in the spleen, indicating that replication of APMV-4 viruses was not extensive in this tissue. Although all the APMV-4 viruses replicated better in ducks than chickens, there was no clear relationship between virus replication and sequence of the F protein cleavage site.

RETRACTED

**Figure 8:** Histopathology and immunohistochemistry in sections of collected tissues from 3-week-old ducks infected with parental and F protein cleavage site mutant APMV-4 viruses. As described in Table 3, ducks were inoculated with each virus (256 HA units) by the combined intranasal and intratracheal routes, and tissue samples were harvested on 4 dpi. The tissues were fixed with formalin and sections were prepared and stained with hematoxylin and eosin for histopathology (A) or with antiserum against the N protein of APMV-4 for immunohistochemistry (B). (A) Histopathological examination of tissue samples revealed similar microscopic findings in parent and mutant APMV-4 viruses. This is illustrated with representative virus, rAPMV-4. The trachea showed mild to moderate lymphocytic tracheitis with mild to moderate multifocal mucosal attenuation and reduction of tracheal mucous glands. Lung sections exhibited moderate to marked multifocal, lymphohistiocytic bronchointerstitial pneumonia with mild to moderate perivascular cuffing in the pulmonary interstitium. Spleen sections showed moderate reactive lymphoid hyperplasia characterized by expansion of the white pulp by reactive lymphocytes and increase size and cell density of lymphoid follicles. (B) The presence of antigen (stained red) was detected for parental and mutant APMV-4 in the epithelial lining of trachea, in the epithelium surrounding the medium and small bronchi of the lungs and in the spleen.

## Discussion

Paramyxovirus infectivity depends on activation of the F protein by proteolytic cleavage by host protease. In the case of NDV, the cleavage site sequence is a major determinant of viral pathogenicity [8], [24], [26]. Virulent NDV strains contain a multibasic cleavage site with a furin motif [RX(R/K)R↓]. In cell culture, this provides for intracellular cleavage without the need for exogenous protease [26]. *In vivo*, these viruses replicate in most cell types and can cause systemic infection. In contrast, the cleavage site sequences of avirulent NDV strains characteristically have one or a few basic residues immediately upstream of the cleavage site in place of a furin cleavage site, thus requiring exogenous protease in cell culture [8], [26]. Replication of avirulent NDV strains is restricted mostly to the respiratory and gastrointestinal tracts, where these extracellular proteases are present. However, some of the other APMV serotypes have incongruities with the NDV paradigm. For example, for a number of the other eight serotypes, the sequence of the cleavage site does not predict whether exogenous protease is needed for growth *in vitro*. For example, the F protein cleavage sites of APMV-2 (PASR↓F), APMV-4 (IQPR↓F) and APMV-7 (PSSR↓F) all contain a single basic residue (R) immediately upstream of the putative cleavage site, but supplementation of exogenous protease (i.e., 10% allantoic fluid) did not enhance virus growth [10], [14], [15]. Thus, for a number of the APMV serotypes, the F cleavage site sequence does not predict the cleavage phenotype *in vitro*. Its contributions to virus replication and pathogenicity *in vivo* remain largely unknown.

RETRACTED

In this study, a reverse genetics system for APMV-4 was developed to investigate the role of the F protein cleavage site in APMV-4 replication and pathogenesis. We constructed a series of mutants with increasing numbers of basic residues, including examples with a furin cleavage site, and evaluated their effects on replication and formation of syncytia *in vitro* as well as replication, tissue tropism, and pathogenicity in chickens and mallard ducks. We were unable to recover mutants containing the cleavage sites of APMV-3 and APMV-5 (RPRGR↓L and KRKKR↓F, respectively), even though the latter was multi-basic and contained the furin motif. However, we readily recovered a mutant containing the cleavage site of NDV strain BC (RRQKR↓F). We noted that this last sequence had a glutamine residue in the -3 position, which typically is the case for NDV strains in general and also is the case for APMV-4. Furthermore, we had previously found that changing this glutamine residue to a basic residue, arginine, in NDV strain BC resulted in virus attenuation in chickens [28]. This indicated that this residue can be important for F protein function in some situations, although it is found in some but not all naturally occurring paramyxovirus F cleavage sequences. We therefore modified the cleavage site sequences of APMV-3 and APMV-5 to contain a glutamine in the -3 positions (RPQGR↓F and KRQKR↓F, respectively) and inserted these sequences into rAPMV-4. These viruses were readily recovered, indicating that this residue indeed was important for APMV-4. This was further confirmed by recovery of three additional mutants containing a glutamine residue in the -3 position.

The six mutant viruses contained 1 to 4 basic residues at their F protein cleavage sites, and in only two cases was a furin motif present (rAPMV-4/Fc type5-Q and rAPMV-4/Fc BC). Nonetheless, none of the mutants required added protease for replication in cell culture, and their replication was not enhanced by added protease. Thus, although a number of these cleavage sites are associated with protease dependence in their respective native viruses (i.e., NDV strain LaSota, SV, and PIV1), all of them became protease independent when transferred into the APMV-4 backbone. However, the ability to form syncytia in cell culture depended on the presence of a furin motif. This was observed most prominently with the mutant containing the cleavage sequence from NDV strain BC (rAPMV-4/Fc BC), and to a lesser extent with the modified site from APMV-5 (rAPMV-4/Fc type5-Q). In contrast, the other cleavage site sequences did not confer syncytium formation in infected cells even after supplementation with allantoic fluid as a source of protease. Furthermore, we confirmed that the presence of a furin site (rAPMV-4/Fc BC and rAPMV-4/Fc type5-Q) can efficiently enhance the F protein cleavage of APMV-4, thus increasing virus replication *in vitro*. This suggests that the enhanced growth was due to increased cell-to-cell spread of the virus associated with the observed syncytium formation. In contrast, the other cleavage site sequences did not confer increased cleavage efficiency and replication *in vitro*. In contrast, evaluation of the pathogenicity of the wild-type and mutant APMV-4 viruses using the ICPI and MDT assays indicated avirulence of APMV-4 [10], [36] without any increase in pathogenicity by any of the mutations. These findings are incongruent with the well-known NDV paradigm, in which the presence of a furin site is a major determinant of virulence [11], [26]. Since the natural host of APMV-4 is not known, it is possible that the F cleavage site of APMV-4 (IQPR↓F), which is not a furin motif, is cleaved efficiently by a protease that is only found in its natural host.

RETRACTED

We investigated whether the avirulence of APMV-4 was due to its inability to replicate in neuronal cells, as assayed using primary neuronal cell cultures as well as inoculation into the brains of 1-day-old chicks followed by quantitation of viral replication. Sporadic expression of APMV-4 antigen in neuronal cells *in vitro* was only observed with the APMV-4 mutant bearing the cleavage site from the neurovirulent NDV strain BC, and compared to the abundant expression of viral antigen observed with the NDV strain BC positive control. Furthermore, all of the parental and mutant APMV-4 viruses, including the one with the NDV BC cleavage site, failed to detectably replicate in neuronal cell cultures *in vitro* or in the brains of chicks inoculated intracerebrally at 1 day of age, in contrast to the abundant replication observed with the NDV strain BC positive control. These results indicate that the avirulence of parental and mutant APMV-4 may be determined, at least in part, by their inability to infect neuronal cells.

For NDV, virus neurotropism depends on the presence of a furin cleavage site, since secretory proteases are unavailable in the brain [37]. However, the present results show that the introduction of a furin cleavage site into the F protein of APMV-4 did not confer neurotropism apart from the limited antigen expression by the rAPMV-4/Fc BC mutant. The general lack of neurotropism by the present rAPMV-4 mutants is reminiscent of our previous study in which the F protein cleavage site sequence of APMV-2 or APMV-7 was changed by reverse genetics into mutants that included ones with furin cleavage sites. In those studies, we made the similar observation that the changes did not increase the neurotropism of APMV-2 or APMV-7 in 1-day-old chicks or 2-week-old chickens [30], [32]. This indicated that, for these three APMV serotypes, the sequence at the F protein cleavage site is not a major determinant of neurotropism. However, in another study, replacement of the complete APMV-2 F protein with that of neurovirulent NDV strain BC was sufficient to confer the neurotropic, neuroinvasive, and neurovirulent phenotypes to APMV-2 [33]. This previous result suggested that the F protein plays an important role in neurotropism, but the present study indicates that this effect does not appear to be determined primarily by the sequence at the F protein cleavage site.

We further evaluated APMV-4 replication in 1-day-old chicks and 2-week-old chickens following inoculation of the respiratory tract. In 1-day-old chicks, the parental viruses and all the mutant APMV-4 viruses were restricted to the trachea and replicated only to low titers. In the 2-week-old chickens, virus replication was detected only sporadically and only in the trachea. However, all of the birds exhibited seroconversion, suggesting that viral infection occurred in each case, but at a low level that often was undetectable by assays for infectious virus. Our recent pathogenicity study with the nine APMV serotypes showed inefficient replication of APMV-4 in chickens [36]. The present results confirm the highly restricted nature of replication of APMV-4, and show that this high level of restriction was not alleviated by the introduction of additional basic residues, including a furin motif, into the F protein cleavage site.

We also evaluated infection of mallard ducks, representing a natural host. The parental and mutant viruses replicated somewhat better in ducks than in chickens. Detection was sporadic for every virus, with virus being detected in the trachea and lungs, and in some cases the spleen, but without inducing any disease. Thus, ducks were more permissive than chickens, but the parental and mutant APMV-4 viruses remained highly restricted and avirulent even in ducks. Detection in the spleen was suggestive of systemic spread, but this was seen sporadically with wild-type rAPMV-4 and several mutants and did not correlate with the presence of a furin cleavage site.

RETRACTED

The present results indicate that, while the introduction of a furin motif into the cleavage site of APMV-4 increased F protein cleavage efficiency, viral replication *in vitro* and conferred the ability to induce syncytia, it did not confer increased replication, tropism, or pathogenesis *in vivo*. Thus, APMV-4 remained highly restricted and avirulent even with the presence of the F protein cleavage site from the neurotropic NDV strain BC. These observations are consistent with previous findings that modification of the F protein cleavage site sequence of APMV-2 and APMV-7 to contain multibasic residues, including furin motifs, did not increase virus pathogenicity in chickens despite their gain of *in vitro* replication and syncytium formation [30], [32]. This indicated that the F protein cleavage site is not a primary determinant or limiting factor to viral virulence for these three serotypes of APMV, indicating incongruity with the well-known NDV paradigm. These results suggest that, for these APMV serotypes to be virulent, changes in other regions of the F protein or in some other viral proteins are necessary. Further characterization of virus replication and pathogenicity using reverse genetics may enhance our understanding of overall APMV pathogenesis.
